# Exercise therapy for prevention of falls in people with Parkinson's disease: A protocol for a randomised controlled trial and economic evaluation

**DOI:** 10.1186/1471-2377-9-4

**Published:** 2009-01-22

**Authors:** Colleen G Canning, Cathie Sherrington, Stephen R Lord, Victor SC Fung, Jacqueline CT Close, Mark D Latt, Kirsten Howard, Natalie E Allen, Sandra D O'Rourke, Susan M Murray

**Affiliations:** 1 Clinical and Rehabilitation Sciences Research Group, Faculty of Health Sciences, The University of Sydney, PO Box 170, Lidcombe, NSW 1825, Australia; 2 Musculoskeletal Division, The George Institute for International Health, The University of Sydney, PO Box M201, Missenden Rd, Sydney, NSW 2050, Australia; 3 Prince of Wales Medical Research Institute, PO Box 82, St Pauls, NSW 2031, Australia; 4 Department of Neurology, Westmead Hospital, Westmead, NSW 2145, Australia; 5 Department of General Geriatric and Rehabilitation Medicine, Royal Prince Alfred Hospital, KGV Buiding, Level 7, Missenden Rd, Camperdown, NSW 2030, Australia; 6 School of Public Health, A27 Edward Ford Bld, The University of Sydney, Sydney, NSW 2006, Australia

## Abstract

**Background:**

People with Parkinson's disease are twice as likely to be recurrent fallers compared to other older people. As these falls have devastating consequences, there is an urgent need to identify and test innovative interventions with the potential to reduce falls in people with Parkinson's disease. The main objective of this randomised controlled trial is to determine whether fall rates can be reduced in people with Parkinson's disease using exercise targeting three potentially remediable risk factors for falls (reduced balance, reduced leg muscle strength and freezing of gait). In addition we will establish the cost effectiveness of the exercise program from the health provider's perspective.

**Methods/Design:**

230 community-dwelling participants with idiopathic Parkinson's disease will be recruited. Eligible participants will also have a history of falls or be identified as being at risk of falls on assessment. Participants will be randomly allocated to a usual-care control group or an intervention group which will undertake weight-bearing balance and strengthening exercises and use cueing strategies to address freezing of gait. The intervention group will choose between the home-based or support group-based mode of the program. Participants in both groups will receive standardized falls prevention advice. The primary outcome measure will be fall rates. Participants will record falls and medical interventions in a diary for the duration of the 6-month intervention period. Secondary measures include the Parkinson's Disease Falls Risk Score, maximal leg muscle strength, standing balance, the Short Physical Performance Battery, freezing of gait, health and well being, habitual physical activity and positive and negative affect schedule.

**Discussion:**

No adequately powered studies have investigated exercise interventions aimed at reducing falls in people with Parkinson's disease. This trial will determine the effectiveness of the exercise intervention in reducing falls and its cost effectiveness. This pragmatic program, if found to be effective, has the potential to be implemented within existing community services.

**Trial registration:**

The protocol for this study is registered with the Australian New Zealand Clinical Trials Registry (ACTRN12608000303347).

## Background

The number of persons with Parkinson's disease over age 50 in Western Europe's five most populous nations was up to 4.6 million in 2005, and this will double to up to 9.3 million by 2030 [1]. Over 100,000 Australians are currently living with Parkinson's disease [2] and in line with estimates from Western Europe this number is also expected to double by 2030 [1]. Since the most common age of onset is 50–60 years and life expectancy is near normal, people with Parkinson's disease suffer the debilitating consequences of the disease over decades.

The mainstay of medical treatment for Parkinson's disease is pharmacological therapy to boost depleted dopamine levels. Despite optimal medication, people with Parkinson's disease living in the community experience frequent and recurrent falls with devastating consequences. Up to 68% of people with Parkinson's disease will fall and up to 46% of people with Parkinson's disease will experience recurrent falls each year [3-6]. These rates are around twice of those in the general older population [6]. In addition, a 12-month prospective study (n = 113) found that 27% of people with Parkinson's disease fell at least once each month and 15% fell at least once a week [3].

Among people with Parkinson disease, as many as 65% of fallers will experience an injury secondary to their falls, 33% will suffer a fracture and 75% of falls will lead to use of a health care service [7]. Falls and related fractures are the most common secondary reason that people with Parkinson's disease are admitted to hospital [8]. These falls have devastating consequences and are accompanied by pain, reduced mobility and unacceptably high levels of caregiver stress. Fear of falling is also greater in community-dwelling people with Parkinson's disease than healthy controls [9]. This results in restriction of activities, compromising quality of life and predisposing to secondary reductions in muscle strength and cardiovascular fitness.

Recently Latt (2006) tested a battery of physiological and clinical variables considered to be potential risk factors for falls in people with Parkinson's disease [3]. These included Parkinson's specific impairments, such as slowness of movement, poor balance, freezing of gait and cognitive impairment as well as age-related impairments, such as reduced lower limb muscle strength. After adjusting for past falls, it was found that freezing of gait, poor balance and lower limb muscle weakness were independent predictors of falls. Therefore, the logical targets for an exercise program designed to reduce falls would be freezing of gait, balance and lower limb muscle strength.

Systematic reviews in the general older population, have found that exercise programs which specifically target balance and lower limb muscle strength are effective in preventing falls [10,11]. In people with Parkinson's disease, lower limb muscle strength and regular exercise are significantly correlated with physical abilities [12-15], therefore highlighting the role of exercise as an appropriate intervention in this population. Exercise has been shown to improve balance [16-18] and strength [18,19] and cueing training [20] has been shown to improve freezing of gait [17] in people with Parkinson's disease. However, no previous randomised controlled trials have investigated an exercise intervention aimed at reducing falls in people with Parkinson's disease by simultaneously targeting all three of these predictors of falls. The Weight-bearing Exercise for Better Balance (WEBB) exercise program has been developed to specifically target poor balance and lower limb muscle weakness for people at risk of falls. The PD-WEBB program used in this study includes progressive weight-bearing balance and strength exercises along with evidence-based cueing strategies to address freezing of gait. (The PD-WEBB program is available from the authors on request).

The primary aim of this randomised controlled trial is to determine the effectiveness of the PD-WEBB exercise program in reducing the rate of falls in people with Parkinson's disease. In addition, we will establish the cost effectiveness of the program from the health provider's perspective and determine the effects of the program on i) risk factors for falls, ii) physical abilities, iii) fear of falling and iv) quality of life.

## Methods

### Design

A prospective, randomised controlled trial will be conducted with 230 community-dwelling participants with Parkinson's disease (Figure 1).

**Figure 1:** **Trial design**.

### Participant selection

To be included in the study participants must meet the following inclusion criteria: (i) a diagnosis of idiopathic Parkinson's disease; (ii) aged 40 years or over; (iii) able to walk independently with or without a walking frame; (iv) fallen at least once in the past 12 months or found to be at risk of falls on assessment; (v) have adapted to their current anti-Parkinsonian medication for at least 2 weeks.

Participants will be excluded if they have a Mini-Mental State Examination score of < 24, or suffer from unstable cardiovascular disease, or suffer from other uncontrolled chronic conditions that would interfere with the safety and conduct of the training and testing protocol or interpretation of the results.

All volunteers will be screened by a physiotherapist. Medical clearance will be required from each participant's medical practitioner to certify him/her as able to participate in moderate-intensity semi-supervised exercise before being accepted into the trial.

The study protocol has been approved by The University of Sydney Human Research Ethics Committee (HREC Number 11-2007/10487), and Sydney West Area Health Service Human Research Ethics Committee (HREC2008/9/4.13 (2865) AU RED 08/WMEAD/250) and written informed consent will be obtained from all participants.

### Measurements and Procedures

All participants will undergo two measurements: one on entry to the study (pre-test) and one after the 6-month intervention period (post-test). All pre-test measures will be assessed prior to randomisation. Cognitive function will be assessed with the Mini Mental State Examination [21]. Measurements will be conducted one hour after each participant's last dose of L-dopa, thus each participant will be tested in their "on" phase.

### Randomization

After completion of the pre-test assessment, participants will be formally entered into the study and randomized to intervention or control groups. Randomization will be stratified by falls history (0–10 falls in the previous 12 months/more than 10 falls in the previous 12 months) using a computer-generated random number schedule with variable block sizes of 2–6. Randomization will be performed centrally by an investigator not involved in recruitment or assessments.

### Intervention Group

#### Program

The intervention group will undertake the PD-WEBB program. This includes a 40–60 min program of progressive balance and lower limb strengthening exercises 3 times a week for 6 months as well as evidence-based cueing strategies to reduce freezing of gait [20]. Participants will have the option to participate in a *support group*-*based *program in which they attend monthly exercise classes conducted by a physiotherapist as well as perform the exercises at home. If they choose this option, the exercises will be updated by the physiotherapist at the class and they will receive two to four home visits by the physiotherapist over the 6 months to ensure that the exercises are performed safely and effectively at home. Participants who choose the *home-based *mode will have eight to ten sessions supervised and progressed by a physiotherapist over the 6 months. These participants will carry out the other sessions independently, following specific written and pictorial instructions provided by the physiotherapist.

#### Exercises

All exercise sessions will include 5 minutes warm-up exercises. The lower limb extensor muscle groups, which act to prevent collapse of the lower limb (hip and knee extensors and ankle plantarflexors) will be targeted with exercises designed to enhance postural control (i. e. balance) and muscle strength. The balance exercises include standing with a decreased base of support, forwards and sideways stepping/walking, and graded reaching activities in standing. Strengthening exercises will include sit-to-stand, forward or lateral step-ups onto a small block, semi squats and heel raises in standing. Resistance for strengthening exercises will be applied using weighted vests in a similar protocol to one which has been successfully used by people with multiple sclerosis in a home-based program [22]. Standard principles governing frequency, volume, duration, intensity and progression of exercise will be applied [23]. Cueing strategies will be used to reduce freezing [17,20,24]. These include identifying appropriate methods of cueing (cognitive, auditory, somatosensory) for each participant and incorporating these cues into everyday activities.

#### Safety

Participants will be instructed how to perform exercises safely with stable supports (such as a table) located nearby for additional support if required. Maintaining safety while exercising will be a prime consideration when level of difficulty of exercises is prescribed and progressed. Participants will be provided with a booklet containing safety precautions, instructions and photographs of exercises for use in exercise sessions at home. In addition, they will be provided with a logbook for recording exercises completed and effects of exercise (e.g. muscle soreness). Any participant who does not demonstrate safety in the independent performance of their exercises after two home visits will be withdrawn from the study. Where appropriate, family members and/or carers, will be encouraged to assist with supervision and performance of the exercise program.

The intervention group will also receive standardised falls prevention advice in the form of a booklet.

### Control group

The control group will receive their usual care from their medical practitioner and community services. In addition, standardised falls prevention advice in the form of a booklet will be provided.

### Outcome measures

The primary outcome measure will be falls:

*Falls *will be assessed by comparing the number of falls in intervention and control groups. The proportion of fallers in each group will also be compared. Falls will be recorded by the use of a "falls diary". All participants will receive monthly calendars on entry to the study, with instructions to record the following events: number of falls, visits by or to nursing and allied health personnel, general practitioner or specialists appointments and hospitalisations. Participants will be asked to return the completed calendar monthly in pre-paid envelopes to the research personnel who are unaware of group allocation. All participants will also be telephoned monthly to record any changes in medications, use of health resources and verify any falls details (including how and where the fall occurred, injuries suffered, medical intervention required and limitations to activity as a result of a fall).

To evaluate the cost effectiveness of the exercise program the following measures will be collected:

*Costs of the intervention: *the costs of implementing the exercise program will be obtained from trial records and research group financial records using actual costs when available. Costs associated with developing and evaluating the exercise program will be excluded from the analysis.

*Costs of health services used for managing fall-related injuries*: use of public and private healthcare resources will be recorded as part of the monthly telephone calls, over the 6-month intervention period.

The secondary outcome measures listed below will be collected on entry to the study and at the end of the 6-month intervention period by an assessor unaware of group allocation. The order of measurements will be standardized. Participants will be instructed not to inform the assessors of their intervention status, and all home exercise equipment will be removed or concealed prior to the post-assessment.

Secondary outcome measures are:

(i) *Parkinson's Disease Falls Risk Score: *Falls risk status will be determined using the Parkinson's disease-specific algorithm developed in our recent large prospective cohort study [3]. This involves weighted contributions from neurological and physiological function measures including gait freezing, impaired balance and lower limb weakness.

(ii) *Maximal muscle strength *of the knee extensor muscles of each leg will be tested using a strain gauge [25].

(iii) *Balance in standing*, using the coordinated stability test which requires participants to accurately adjust their position in a steady and coordinated manner when their centre of mass is near the limits of their base of support [26].

(iv) *Short Physical Performance Battery*, including tests of walking, balanced standing and sit to stand [27].

(v) *Freezing of gait*, using the Freezing of Gait Questionnaire [28].

(vi) *Falls Efficacy Scale International*, a falls efficacy questionnaire [29].

(vii) *Health and Well-being*, using the SF12v2™.

(viii) *Habitual Physical Activity Questionnaire *to quantify the type and amount of regular physical activity.

(ix) *PDQ-39*, a Parkinson's disease specific quality of life questionnaire [30].

(x)* Positive and Negative Affect*, using the Positive and Negative Affect Schedule (PANAS) [31].

Adverse events (defined as a significant injury or medical event that causes the participant to seek attention from a health professional or limit their activities) will be monitored and recorded throughout the study during the monthly telephone calls to each participant.

### Statistical analysis

The number of falls per person-year will be analysed using negative binomial regression to estimate the difference in fall rates between the two groups, adjusted for previous multiple faller status and other confounding variables if required [32]. The proportion of fallers between groups will be compared using the relative risk statistic. Between-group comparisons of final test performance for the continuously-scored outcome measures will be made using General Linear Models (ANCOVA) controlled for pre-test performance. Baseline continuously-scored data will be compared between groups using the student t-test. Ordinally-scored data will be analysed for between group differences using the non-parametric Mann Whitney U statistic. An intention-to-treat approach will be used for all analyses.

Economic analysis will be undertaken in the manner used in previous falls prevention studies [33,34]. The total costs in intervention and control groups (including the cost of the exercise program, and costs of health and community service contacts) and falls rates, will be used to calculate an incremental cost per fall prevented in the intervention group compared with the control group. Bootstrapping will be used to estimate a distribution around costs and health outcomes and to calculate confidence intervals around the cost-effectiveness ratio; one-way sensitivity analyses will be conducted around key parameters.

### Sample size

As fall rates will be compared between groups using incident rate ratios (IRR) from negative bionomial regression models [32] we conducted an analysis of statistical power using the nbpower command in the STATA software package. A total of 230 participants (115 per group) will be required to provide 80% power to detect as significant, at the 5% level, a 30% lower rate of falls for exercise subjects than control subjects (i. e. IRR = 0.70). We assumed the control group rate of falls would be 1 fall/person month over the 6-month follow-up period, a conservative estimate as the prospective cohort study [3] reported a falls rate of 1.6 falls/person month in a 12-month follow up of 113 people with PD.

The sample size of 230 will also be sufficient to detect between-group differences of 23% of control group values in the coordinated stability (balance) measure (assuming a control group mean of 18 and SD of 14) and 11% for knee extension strength (assuming a control group value of 16 kg and SD of 6). Both calculations are based on values found among fallers with PD [3] assuming 80% power of a two-sided test at the 5% level, a correlation between pre-and post measures of 0.7, and 15% dropouts.

## Discussion

There is an urgent need to identify cost-effective evidence-based interventions for reducing falls and related injuries in people with Parkinson's disease. To date, no adequately-powered studies have investigated exercise interventions aimed at reducing falls in people with Parkinson's disease. Only three randomised controlled trials have reported falls as outcomes. One study found a 38% (rate ratio = 0.62) reduction in rate of falling from a fully-supervised 8-week program of treadmill walking but was clearly under-powered (n = 18, 95% CI of RR 0.26 to 1.48, calculated by CS from published data) [35]. Another reported improved balance, walking and confidence in walking, and a non-significant 40% (odds ratio = 1.40) increase in risk of falling following a 3-week home-based program of rhythmical cueing of walking [17] (95% CI 0.63 to 3.1). The only study which targeted fallers [16] investigated a 6-week home-based program of multi-facetted exercise and showed promising results on balance and a non-significant, but 26% reduced risk of falls (risk ratio for repeat falls at 8 weeks = 0.74, 95% CI 0.47 to 1.15, calculated by CS from published data). A statistically and clinically beneficial reduction in falls risk might have become apparent if the interventions had been of longer duration.

The PD-WEBB program has been designed for falls prevention and so includes high challenge, yet safe, progressive balance exercises targeting standing balance and walking as well as progressive moderate to high intensity leg strengthening exercises with resistance applied using weighted vests. As different individuals have different preferences for exercise, participants who are randomly allocated to the exercise group will have the option to perform the 6-month program of exercises entirely at home (home-based mode) or in association with their Parkinson's support group (support group-based mode) with an additional home exercise program. Both modes of delivery incorporate semi-supervision by a physiotherapist and are designed to be individually tailored. The randomized controlled trial [17] which has addressed freezing (the RESCUE trial) using cued walking practice found no overall effect on freezing, but a significant effect in a subgroup of freezers. Therefore our exercise intervention will incorporate cueing strategies for overcoming freezing [17,20,24] as well as balance and strength exercises.

We will investigate the effect of the PD-WEBB program in people with Parkinson's disease using a randomized controlled trial incorporating the features known to reduce bias (i. e. concealed random allocation to groups, blinded outcome assessment and intention to treat analysis) and large enough to detect any effect of the intervention on fall rates. This project will determine the effectiveness of the exercise intervention in reducing falls, but will also determine the cost effectiveness of the intervention. This program, if found to be effective, has the potential to be implemented at a reasonable and sustainable cost within existing community services. Any reduction in falls for people with Parkinson's disease will reduce the personal and financial costs to individuals with Parkinson's disease, their families, health care resources and the community.

## Competing interests

The authors declare that they have no competing interests.

## Authors' contributions

CGC, CS, SRL, VSCF, JCTC and MDL conceived the idea and obtained funding for the study. All authors contributed to the design and development of the trial protocol. CGC and SDO drafted the manuscript. All authors critically reviewed the manuscript and approved the final manuscript.

## Pre-publication history

The pre-publication history for this paper can be accessed here:


